This article has been retracted.

# Improved Capsule Network Optimization Hierarchical Convolution Algorithm for Mental Health Recognition

**DOI:** 10.1155/2022/5396840

**Published:** 2022-04-09

**Authors:** Tapas Bhowmik, Rohini A. Bhusnurmath, Deepti Sahu, Jyotsna, K. Suresh Babu, Abdullah Alqahtani

**Affiliations:** ^1^Canadian University of Bangladesh, Bangladesh; ^2^Department of Computer Science, Akkamahadevi Women's University, Vijayapura, Karnataka, India; ^3^Department of Computer Science and Engineering, Sharda University, Greater Noida, India; ^4^Department of Biochemistry, Symbiosis Medical College for Women, Symbiosis International (Deemed University), Pune, India; ^5^Department of Computer Science, College of Computer Science, King Khalid University, Abha, Saudi Arabia

## Abstract

To address the shortcomings of standard convolutional neural networks (CNNs), the model structure is complex, the training period is lengthy, and the data processing technique is single. A modified capsule network is presented to optimize hierarchical convolution—the algorithm for identifying mental health conditions. To begin, two types of data processing are performed on the original vibration data: wavelet noise reduction and wavelet packet noise reduction; this retains more valuable information for mental health identification in the original signal; secondly, the CNN employs the concept of hierarchical convolution, and three distinct scaled convolution kernels are utilized to extract features from numerous angles; ultimately, the convolution kernel's extracted features are fed into the pruning strategy's capsule network for mental health diagnosis. The enhanced capsule network has the potential to significantly speed up mental health identification while maintaining accuracy. It is time to address the issue of the CNN structure being too complex and the recognition impact being inadequate. The experimental findings indicate that the suggested algorithm achieves a high level of recognition accuracy while consuming a small amount of time.

## 1. Introduction

With the continuous development of industrial applications, factory equipment tends to be large-scale and intelligent, and safety issues have always been concerned. For example, rolling bearings are an indispensable key component of rotating equipment. Due to their long working hours and large workloads, there will inevitably be damage to parts, which will affect the efficiency of the factory in light, and will have a particular impact on the life safety of operators. In medicine, “mental health” refers to a state of being sick. Therefore, considering that bearing failures are not formed instantly, the “mental health” state in medicine can be used to characterize the running state of bearings with the disease. Of course, the equipment will not fail immediately, but if it continues to run without updating parts, it will bring serious consequences. Hence, the health status monitoring of “mental health” equipment is of great economic and safety significance [1–4]. The optimized hierarchical convolution mental health detection algorithm is used to collect characteristics from various angles; the retrieved characteristics from the convolutional network are then fed into the pruning strategy's capsule network for mental health diagnosis. The improved capsule network has the ability to dramatically accelerate mental health detection while preserving efficiency.

Given the ongoing research by artificial intelligence researchers into defect detection and diagnosis technology, the identification of bearing mental health state has advanced to a relatively mature stage. With the advancement of deep learning, an end-to-end deep learning model-convolutional neural network combination has been widely adopted and applied in a variety of disciplines. This research proposes to improve the capsule network to optimize the layering CNN's mental health recognition algorithm. Although numerous professionals and academics have applied deep learning knowledge to the mental health identification of bearings and produced favorable mental health identification outcomes, the technology is still in its infancy. As a result, it requires ongoing education and exploration [5–7].

Convolutional neural networks were the fundamental models employed in fault diagnosis by two international scientists in 2019. Marchisio et al. converted one-dimensional vibration signals to two-dimensional images, utilizing the superiority of convolutional neural networks for image classification, and achieved excellent recognition results with robustness, the ability to withstand noisy environments, and the absence of a feature extraction step [8]. The SVM is a supervised learning technique that can be used in both classification and regression. Although we may also argue recurrent difficulties, categorization is the perfect suited. For big data sets, the SVM method is ineffective. Whenever the data set contains additional noise, such as identical target classes, SVM sometimes does not perform well. Islam adopts the convolutional neural network as a starting point and presents a more adaptable deep convolutional neural network. It provides azimuth health status information using a two-dimensional visualization of the original acoustic emission signal and the discrete wavelet transform as a 2D visualization tool. The evaluation metrics accurately depict each fault condition, and beneficial bearing fault characteristics are learned automatically [9].

Although the convolutional neural network (CNN) has achieved good results in specific fields, there are still problems such as reducing the scalar activity of some neurons during feature extraction and the loss of detailed spatial information in the pooling layer. In 2021, the capsule network proposed by Byerly and Kalganova solved the problem of CNN [10]. Given the advantages of capsule networks, many experts in fault diagnosis have also begun to conduct research.

Scholars such as Zhu use a short-time Fourier transform to convert the original signal to a two-dimensional image. Inception module and regression branch are used to input the two-dimensional image into a new capsule network inspired by the dynamic routing capsule network. The capsule's length corresponds to the associated fault type. The other two components regress the damage size of the tablet using the most extended tablet, while the other branch reconstructs the input graph. Experiments demonstrate that the suggested model is very generalizable and has high recognition accuracy. [11]. Chen et al. suggested a stochastic delta rule deep capsule network to overcome the limitations of raw vibration signals in terms of workload change and noise effects. The suggested model has a deep structure and pooling operations do not require a one-dimensional convolution layer. The capsule's higher-level features can be extracted, and the capsule's receiving region can be extended. The original vibration signal is used as the input, and noise is fed into the first wide layer to enhance the antinoise capability. Experiments demonstrate that this approach works under a variety of load conditions. Additionally, it obtains a high degree of accuracy [12].

The researchers mentioned above have designed deep convolutional neural networks to obtain high accuracy. The model structure is deep and complex. However, scholars using capsule networks have not proposed a solution to the redundancy of internal features of capsules. On this basis, this paper presents an improved capsule network to optimize the mental health recognition model of hierarchical CNN. The original vibration data is input into the hierarchical CNN after wavelet noise reduction and wavelet packet noise reduction for feature extraction and then input into the improved capsule network for feature extraction. Mental health recognition reduces feature redundancy in capsule vector, and the proposed model speeds up the recognition time of mental health when recognition accuracy.

The present article has been planned into various sections.  Section 1 describes the introduction of the proposed research, Section 2 puts light on convolutional neural network, the capsule network is describe in Section 3, the experimental setup and result analysis is describe in Section 4, and finally, Section 5 portrays the conclusion and possible future works based on the proposed framework.

## 2. Convolutional Neural Network

Yann LeCun proposed a convolutional neural network (CNN) in 1989. It was initially used to recognize handwritten digits, and then, it was widely used in the field of image processing. Since it does not require preprocessing for feature extraction, the original input image can be directly output, so it is widely used. This processing mode is called an “end-to-end” processing mode [13, 14]. A schematic diagram of a simple CNN structure is shown in Figure 1.

In a typical convolutional neural network system, several types of coverings have distinct roles and include convolutionary layers, pooling layers, and fully connected layers. A key part of CNN is the convolution layer. It performs the convolution on the local area of the input signal using the convolution kernel. The input data from the preceding layer is convolved using the convolution kernel's sliding process, and the convolution operation is done. The sharing of weight is the most critical aspect. An equation describing the convolution process is as follows:

(1) $$\begin{array}{c} X_{j}^{l}=f\left(\overset{N}{\underset{i=1}{\sum }}x_{i}^{l-1}.{\text{k}}_{ij}^{l}+b_{j}^{l}\right), \end{array}$$

where *N* is the kernel tree at layer *l* − 1, *x*_*i*_^*l*−1^ is the input of the kernel, *x*_*j*_^*l*^ is the output of the grain, *k* and *b* are the corresponding kernel and bias, and *f*() is the nonlinearity. The activation function is used to improve the expressiveness of features through nonlinear operations.

The pooling layer is used to minimize the size of the network parameters and ensure translation invariance. Mean pooling and maximum pooling are the most often used pooling functions [15]. Mean pooling outputs the mean value inside the convolution kernel, whereas maximum pooling outputs the entire value within the convolution kernel. Equations (2) and (3) illustrate the formulas:

(2) $$\begin{array}{c} P_{l+1}^{i}\left(j\right)=\frac{1}{w}\overset{jw}{\underset{t=\left(j-1\right)w+1}{\sum }}a_{l}^{i}\left(\text{t}\right), \end{array}$$

(3) $$\begin{array}{c} P_{l+1}^{i}\left(j\right)=\underset{\left(j-1\right)w+1⩽t⩽jw}{\max}\left\{a_{l}^{i}\left(t\right)\right\}. \end{array}$$

Among them, *w* denotes the pooling width, *P*_*l*+1_^*i*^(*j*) is the value associated with the neuron in layer *l* + 1, and *a*_*l*_^*i*^(*t*) denotes the activation value associated with the neuron in the *i*th feature plane of the *l*th layer.

Classification is accomplished by the use of fully connected layers. The specific operation is as follows: first, the neurons in the preceding layer are formed into a one-dimensional feature vector, and then, the input and output are connected completely [16].

## 3. Capsule Network

Capsule network (capsule network, CapsNet) mainly includes a convolutional layer, main cap layer, digital cap layer, and decoder. In the capsule network, dynamic routing is applied continuously to update the parameters [17, 18]. Its model the diagram is shown in Figure 2.

The structure of the capsule network consists of four parts [19, 20]:

1. *Convolution Layer*. It simply processes the input data to extract features. The convolution formula is shown in formula (1). The convolution operation of the capsule network is similar to that of the convolution neural network.
2. *Main Cap Layer.* Different characterizations are divided into vector-valued capsules by this function. This layer is capable of capturing the input's instantiation parameters, which may be written as formula (4):

(4) $$\begin{array}{c} u^{l\left(i,j\right)}=f_{s}\left(\begin{array}{c} f_{a}\left(z_{1}^{l\left(i,j\right)}\right)\\ f_{a}\left(z_{2}^{l\left(i,j\right)}\right)\\ \cdots \\ f_{a}\left(z_{m}^{l\left(i,j\right)}\right) \end{array}\right)=f_{s}\left(\begin{array}{c} f_{a}\left(K_{1i}^{l}.x^{l\left(r^{j}\right)}\right)\\ f_{a}\left(K_{2i}^{l}.x^{l\left(r^{j}\right)}\right)\\ \cdots \\ f_{a}\left(K_{mi}^{l}.x^{l\left(r^{j}\right)}\right) \end{array}\right), \end{array}$$

where *u*^*l*(*i*, *j*)^ is the central capsule, *f*_*a*_(*z*_*m*_^*l*(*i*, *j*)^) is the activation output of the convolutional layer, and *f*_*s*_ represents the “squeeze” function.

(3) *Digital Cap Layer.* This layer mainly applies compression and dynamic routing. After one “squeeze” operation and three dynamic routing algorithms, the results are output to the classification.

Since the length represents the probability of the capsule, it is necessary to compress it in the range of 0-1, so there is a “squeeze” function as shown in formula (5):

(5) $$\begin{array}{c} v_{j}=\frac{{\left\|s_{j}\right\|}^{2}}{1+{\left\|s_{j}\right\|}^{2}}\frac{s_{j}}{\left\|s_{j}\right\|}, \end{array}$$

where *s*_*j*_ is the input of the “squeeze” function and *v*_*j*_ is the output of the “squeeze” function. The length can be squeezed between 0 and 1 through the “squeeze” function, *s*_*j*_/∣|*s*_*j*_|∣ represents the direction, and ‖*s*_*j*_‖^2^/1 + ‖*s*_*j*_‖^2^ denotes the zoom factor so that the directional features can be well preserved to higher-level capsules.

Dynamic routing is a continuously updated process, including the following:

(6) $$\begin{array}{c} s_{j}=\underset{i}{\sum }c_{ij}u_{j/i}, \end{array}$$

where *u*_*j*/*i*_ is the prediction vector, *c*_*ij*_ is the coupling coefficient, and ∑_*i*_*c*_*ij*_=1.

The Softmax function determines the coupling coefficient:

(7) $$\begin{array}{c} c_{ij}=\frac{\exp\left(b_{ij}\right)}{\sum_{j}\exp\left(b_{ij}\right)}, \end{array}$$

where *b*_*ij*_ is the predicted *u*_*j*/*i*_ coupled log prior probability with the advanced capsule *s*_*j*_.

(8) $$\begin{array}{c} \frac{u_{j}}{i}=W_{ij}.u_{i}, \end{array}$$

where *u*_*i*_ is the *i*th input capsule and *W*_*ij*_ is the weight matrix.

The *b*_*ij*_ formula is shown in formula (9):

(9) $$\begin{array}{c} b_{ij}⟵b_{ij}+\frac{u_{j}}{i}.v_{j}, \end{array}$$

where *u*_*j*/*i*_.*v*_*j*_ corresponds to the log-likelihood between capsules *u*_*j*/*i*_ and *v*_*j*_.

The above Equations (5)–(9) are the dynamic routing update process, and completing the dynamic routing process also completes the parameter update between the two capsule layers.

(4) *Classification Layer*. It is used to classify the final output results.

## 4. Experimental Setup and Result Analysis

The acquisition device, which consists of a motor, torque sensor/encoder, dynamometer, and control electronics, introduces a single point fault into the bearing under test, with a diameter of 0.007 in, and collects vibration data using an accelerometer mounted on the drive end of the motor housing. The vibration data collected is the actual measured data required for the experiment, with a sampling frequency of 12 kHz. Due to the fact that numerous researchers have standardized and recognized the data acquired under this setting, it possesses a high degree of resilience. This data is utilized in this paper to demonstrate the algorithm's performance, and the specific parameters are listed in Table 1.

The model proposed in this paper selects two data preprocessing methods to work together, namely, wavelet noise reduction and wavelet packet noise reduction. The wavelet noise reduction is a statically representation that divides a digital signals or performance into distinct scale elements [21]. Every scale constituent may generally be assigned a frequency range. Both the method retains more valuable information for mental health identification in the original signal.

The wavelet denoising parameters chosen in this paper are as follows: the threshold value is “figure,” the hard threshold value, the number of decomposition layers is 3, and the wavelet basis function is “sym4.” The wavelet packet denoising parameters are hard threshold, decomposition layers are 3, and the wavelet basis function is “db4.” The point is in the form of a fixed point, and its formula is shown in formula (10):

(10) $$\begin{array}{c} \text{th}=\text{sqrt}\left(2\times \log\;n\right), \end{array}$$

where *n* is the signal length.

To improve the model's generalization ability, the idea of reference [13] is used to make a training sample set by sliding window, and the original signal is overlapped to enhance the data set. Selecting the sliding window size as 3000 and the offset as 300, 16 data sets with different loads and states can produce 10,388 data sets for experiments, including 8,656 training sets and 1732 test sets, and the ratio is 5 : 1.

To speed up the training and ensure the model's generalization ability, this paper adopts the batch processing method. Although using a large batch_size will shorten the training data set time, the problem is that the accuracy needs to be the same as when the batch_size is small. Accuracy may take a lot of time, so when batch_size increases to a specific value, the time will be the shortest. The optimal accuracy will be achieved when it reaches a particular matter. To choose a suitable batch_size, the experimental results are shown in Table 2.

It can be seen from the data in Table 2 that when the batch size ≥ 200, with the decrease of the batch size value, the training time continues to increase, the cycle to reach the highest mental health recognition rate is gradually shortened, and the accuracy rate is also continuously improved; the loss value is also decreasing. When the batch size is 100, the cycle to reach the best mental health recognition is shortened, and the loss value is lower. When the batch size is less than 50, the training time is vastly improved, but the accuracy is not improved.

They are not considered. When the batch size is 100 and 200, respectively, although the recognition accuracy is comparable, the loss value and the optimal recognition cycle achieve better results when the batch size is 100. Compared with the time spent, the accuracy of the model is guaranteed. As a principle, 100 is finally selected as the batch size value of this article.

The performance of the mental health identification algorithm proposed in this paper to optimize the hierarchical CNN by improving the capsule network depends mainly on the size of the convolution kernel, the convolution step size, and the coupling coefficient threshold of the pruning. The improved capsule network has the ability to considerably improve mental health detection speed while preserving accuracy. It is time to fix the problem of the CNN structure being extremely complicated and the identification impact being insufficient. This study recommends that the capsule network be improved in order to enhance the multilayer CNN's mental health identification algorithm. In addition, recognition results can have a significant impact. The detailed parameters of the mental health identification model are shown in Table 3.

The structural parameters of the mental health recognition model are described in detail in Table 3. The selected optimizer is the Adam optimizer with a small memory footprint and efficient calculation of an adaptive learning rate. The activation function is ReLU, the learning rate is 0.001, and the loss function is average square error.

The threshold value of the pruning operation is also the parameter to be selected in the experiment. The threshold value will directly affect the accuracy of the final experimental result. When the coupling coefficient is too large, the accuracy rate will decrease. Otherwise, pruning will not shorten the training time—the goal of. The relationship between the accuracy of mental health recognition and the pruning threshold is shown in Figure 3.

It can be seen from Figure 3 that when the pruning threshold of the coupling coefficient decreases, the recognition accuracy increases. When the coupling coefficient threshold reaches the best value after 0.02 and tends to be stable and pays special attention to the change of time during the experiment when the threshold value gradually decreases, the time difference of mental health identification is not significant, so the accuracy rate is the selected threshold value. For the main criterion, the final pruning threshold chosen is 0.02.

The selection of specific model structural parameters and coupling coefficients has been introduced in above paragraph. After transforming the dimensions of the original data and inputting it into the network model, the accuracy of mental health identification can be obtained. The accuracy of the experiment is shown in Table 4.

As illustrated in Table 4, the CNN's mental health recognition algorithm is optimized using a capsule network to attain a higher level of recognition. The efficiency of the mental health detection technique described in this study to improve the hierarchical CNN by upgrading the capsule network is mostly affected by the size of the convolution kernel, the convolution step size, and the pruning coupling coefficient threshold. The upgraded capsule network's recognition accuracy is comparable to that of the original capsule network. There is feature redundancy; regardless of whether the content stated by the bottom capsule and the high-level pill are consistent, the update with dynamic routing policy will be performed. When implementing the pruning method, set the coupling coefficient below a certain threshold to 0, as this portion of the coupling coefficient has no effect on the final recognition result. When the pruning approach is employed, the capsule vector's feature redundancy is decreased. It will have no effect on the accuracy of recognition. Although the figures above demonstrate unequivocally that the upgraded CapsNet described in this paper has a higher recognition rate, it is not significantly different from the original CapsNet. As a result, the time required for mental health recognition of the proposed model is compared to the time required for three mental health credits.  Table 5 summarizes the findings.

Table 5 shows the time comparison before and after the improvement of the algorithm. The results of the first three experiments are selected for intermediate processing. The average time for mental health identification using the original CapsNet is 4.54 s, and the average time for mental health identification using the improved CapsNet is 3.25 s. It can be seen that the recognition time of the enhanced capsule network is 1.29 s faster than that of the original capsule network. It can be seen that the algorithm in this paper has accelerated the recognition time while ensuring accuracy. To verify the effectiveness of the pruning strategy proposed in this paper, special attention is paid to the changes in pruning parameters. The parameters to be trained for the entire model are 2,344,340. When the pruning threshold changes, the pruning parameters are shown in Table 6.

It can be seen from Table 6 that when the pruning threshold is set to 0.02, the number of pruning parameters is 612,648, which can verify the effectiveness of the algorithm in this paper. The recognition accuracy of the algorithm in this paper and the algorithms proposed by scholars in recent years are compared, as shown in Table 7 and Figures 4 and 5.

As demonstrated in Table 7, the enhanced capsule network optimized hierarchical convolutional mental health detection method developed in this article outperforms the weighted permutation entropy-filter & wrapper extreme learning machine (WPE-FWELM), and the improved chicken swarm optimization RBF neural network (GCSO RBFNN, growth chicken swarm optimization-radial basis function neural network) improves recognition accuracy by 7.58 percent and 5.77 percent, respectively. In terms of recognition time, the WPE-FWELM and GCSO-RBFNN algorithms take 200 samples to recognize.

The algorithm described in this work has a recognition time of 3000 samples, and the time required acknowledging a single signal with a length of 3000 is around 1.876 ms, indicating that the mental health recognition algorithm provided in this paper is effective.

Simultaneously, to demonstrate the algorithm's effectiveness, it is compared to the mental health recognition algorithm, whose fundamental model is CNN, as shown in Table 8 and Figure 6.

The proposed improved capsule network optimized hierarchical convolution mental health detection algorithm is compared to a classic convolution neural network with a Softmax classifier and a convolution neural network with a support vector machine (SVM) classifier in Table 8. The comparison of proposed model and previous models on the basis of training and testing time is shown in Figures 7 and 8.

By contrast, conventional convolutional neural network models employ three convolutional layers and three pooling layers. As can be seen, the recognition accuracy of the algorithm in this paper is improved by 1.21 percentage points and 0.10 percentage points, respectively, when compared to the other two traditional CNNs; in terms of recognition time, although the recognition time in this paper is relatively high due to the nature of the data used, the processing method is a sliding window, and the test time is the amount of time required to identify 1732 data sets totaling 3000 bytes. The classic convolution neural networks is better than Softmax classifier in terms of work efficiency. If we compare SVM with CNN, we find that the SVM and neural network may establish a classification function by mapping the incoming data to a higher dimensional space. In the case of SVM, kernel techniques are used, but in the case of neural networks, semiactivation values are used. The time required to identify a single signal with a 3000 is around 1.876 milliseconds. As can be observed, the recognition time is shorter, demonstrating the effectiveness of the proposed mental health recognition algorithms.

## 5. Conclusion

Aiming at the problems that traditional CNN needs to stack convolutional layers continuously and pooling layers to obtain high accuracy, the data processing method is single, and CNN cannot identify the relationship between the part and the whole well; this paper proposes to improve the capsule network to optimize the layering CNN's mental health recognition algorithm. In this research, the authors have used improved capsule network to optimize the mental health recognition model of hierarchical CNN. The improved capsule network has the ability to considerably improve mental health detection speed while preserving accuracy. Since the capsule network uses a dynamic routing algorithm to update the parameter fees when a pruning strategy and a dynamic routing strategy of parameter correction are proposed to speed up the updating process of the dynamic routing algorithm, experiments show that the algorithm in this paper can accurately identify the mental health state of bearings. Still, this paper is only for bearing experimental data, and further experiments are needed for other objects such as motors and fans, and the transfer learning ability is weak. This research will very helpful in future studies. The results show that the proposed algorithm obtains a high level of recognition accuracy rate while consuming a small amount of time. At the same time, the bearing mental health diagnosis proposed in this paper is offline, and real-time mental health identification research and migration model research can be considered in the future.

## Figures and Tables

**Figure 1:** Schematic diagram of CNN.

**Figure 2:** Capsule network.

**Figure 3:** Selection of pruning threshold.

**Figure 4:** Comparison of accuracy of proposed model.

**Figure 5:** Comparison of time taken by proposed model.

**Figure 6:** Comparison of average accuracy of proposed algorithm.

**Figure 7:** Comparison of training time of proposed algorithm.

**Figure 8:** Comparison of test time of proposed algorithm.

**Table 1:** Experimental device parameters.

Bearing status	Load/HP	Fault diameter/in	Speed (/r/min)	Label
Normal	0	None	1797	X97
	1	None	1772	X98
	2	None	1750	X99
	3	None	1730	X100
Inner ring failure	0	0.007	1797	X105
	1	0.007	1772	X106
	2	0.007	1750	X107
	3	0.007	1730	X108
Ball failure	0	0.007	1797	X118
	1	0.007	1772	X119
	2	0.007	1750	X120
	3	0.007	1730	X121
Outer ring failure	0	0.007	1797	X130
	1	0.007	1772	X131
	2	0.007	1750	X132
	3	0.007	1730	X133

**Table 2:** Selection of batch_size.

Batch_size	Cycle	Time/s	Accuracy >99% cycle	Accuracy/%	Loss
500	18	215	8	99.93	0.04834
400	22	223	7	99.95	0.04201
300	29	259	7	99.95	0.03967
250	35	265	6	99.96	0.03742
200	44	277	4	99.96	0.03114
150	58	284	5	99.96	0.03448
100	87	296	3	99.96	0.02930
50	174	345	4	99.95	0.02984
20	433	535	3	99.96	0.02233
10	867	671	3	99.96	0.02346
5	1732	1042	2	99.96	0.01993

**Table 3:** Structural parameters of mental health identification model.

Network layer	Convolution kernel size/stride	Number	Number of outputs/channels	Whether to zero-fill
Conv1	5 × 1/2 × 1	4	1498 × 1/4	N
Concat	—/—	-	1498 × 1/8	-
Conv2	5 × 1/2 × 1	4	747 × 1/4	N
Conv1 × 1	1 × 1/1 × 1	4	747 × 1/4	N
Conv3 × 1	3 × 1/1 × 1	4	747 × 1/4	Y
Conv5 × 1	5 × 1/2 × 1	4	747 × 1/4	Y
Concat	—/—	—/—	747 × 1/12	-
Conv3	3 × 1/1 × 1	4	745 × 1/4	N
PrimaryCap	5 × 1/2 × 1	8	371 × 1/32	N
DigitCaps	—/—	—/—	4/16	-
Length (output)	—/—	—/—	4/—	-

**Table 4:** Mental health recognition accuracy.

Number of experiments	Original CapsNet	Improve CapsNet
The first time	99.95	99.96
The second time	99.95	99.95
The third time	99.97	99.97
Mean	99.96	99.96

**Table 5:** Mental health identification time.

Number of experiments	Original CapsNet	Improve CapsNet
The first time	4.60	3.27
The second time	4.08	3.24
The third time	4.94	3.24
Mean	4.54	3.25

**Table 6:** Changes of pruning parameters.

Pruning threshold	Pruning parameters
0.01	373,181
0.02	612,648
0.03	711,706
0.04	743,791
0.05	753,453

**Table 7:** Accuracy comparison.

Algorithm	Average accuracy/%	Time/s
WPE-FWELM	92.38	0.4267
GCSO-RBFNN	94.19	0.5586
Proposed algorithm	99.96	3.2500

**Table 8:** Comparison with the basic model of CNN.

Algorithm	Average accuracy	Training time (sec)	Test time (sec)
CNN-Softmax	98.75	248	0.279
CNN-SVM	99.86	230	0.187
Algorithm	99.96	296	3.250

## Data Availability

The data shall be made available on request.

## References

[1] Liao W., Chen J., Liu Q., Zhu R., Song L., Yang Z. (2021). Data-driven reactive power optimization for distribution networks using capsule networks. *Journal of Modern Power Systems and Clean Energy*.

[2] Chiadika O. D. -M., Li M., Choi J. Improving training time in capsule neural network.

[3] Topçu M., Dede A., Eken S., Sayar A. Multilabel remote sensing image classification with capsule networks.

[4] Marchisio A., Bussolino B., Colucci A. FasTrCaps: an integrated framework for fast yet accurate training of capsule networks.

[5] Marchisio A., Massa A., Mrazek V., Bussolino B., Martina M., Shafique M. NASCaps: a framework for neural architecture search to optimize the accuracy and hardware efficiency of convolutional capsule networks.

[6] Joseph Z., Nyirenda C. Deepfake detection using a two-stream capsule network.

[7] Sergeyev Y. D., Kvasov D. E., Mukhametzhanov M. S. A generator of multiextremal test classes with known solutions for black-box constrained global optimization. *IEEE Transactions on Evolutionary Computation*.

[8] Marchisio A., Mrazek V., Hanif M. A., Shafique M. (2021). FEECA: design space exploration for low-latency and energy-efficient capsule network accelerators. *in IEEE Transactions on Very Large Scale Integration (VLSI) Systems*.

[9] Kurtakoti A. U., Chickerur S. Steady flow approximation using capsule neural networks.

[10] Byerly A., Kalganova T. (2021). Homogeneous vector capsules enable adaptive gradient descent in convolutional neural networks. *IEEE Access*.

[11] Kakillioglu B., Ren A., Wang Y., Velipasalar S. (2020). 3D capsule networks for object classification with weight pruning. *IEEE Access*.

[12] Ajaz F., Naseem M., Sharma S., Shabaz M., Dhiman G. (2022). COVID-19: challenges and its technological solutions using IoT. *Current Medical Imaging Reviews*.

[13] Ghozali M. T., Satibi S., Ikawati Z., Lazuardi L. (2021). Asthma self-management app for Indonesian asthmatics: a patient-centered design. *Computer Methods and Programs in Biomedicine*.

[14] Heidarian S., Afshar P., Enshaei N. Wso-Caps: diagnosis of lung infection from low and ultra-lowdose CT scans using capsule networks and windowsetting optimization.

[15] Gagana B., Athri H. A. U., Natarajan S. Activation function optimizations for capsule networks.

[16] Roland G., Kumaraperumal S., Kumar S., Gupta A., das Afzal S., Suryakumar M. (2021). PCA (principal component analysis) approach towards identifying the factors determining the medication behavior of Indian patients: an empirical study. *Tobacco Regulatory Science*.

[17] Shang Y., Xu N., Jin Z., Yao X. Capsule network based on self-attention mechanism.

[18] Luo L., Wang M., Song X., Guo S., Chu W., Tan J. Polyphonic sound event detection based on CapsNet-RNN and post processing optimization.

[19] Fontana R., Mulana F., Cavallotti C. (2017). An innovative wireless endoscopic capsule with spherical shape. *IEEE Transactions on Biomedical Circuits and Systems*.

[20] Patel K., Hassan I. U. Identifying fake news with various machine learning model.

[21] Bharti R., Khamparia A., Shabaz M., Dhiman G., Pande S., Singh P. (2021). Prediction of heart disease using a combination of machine learning and deep learning. *Computational Intelligence and Neuroscience*.

